# Detangling PPI networks to uncover functionally meaningful clusters

**DOI:** 10.1186/s12918-018-0550-5

**Published:** 2018-03-21

**Authors:** Sarah Hall-Swan, Jake Crawford, Rebecca Newman, Lenore J. Cowen

**Affiliations:** Department of Computer Science, Tufts University, Medford, 02155 MA USA

**Keywords:** PPI networks, Protein function prediction, Community detection, Diffusion state distance

## Abstract

**Background:**

Decomposing a protein-protein interaction network (PPI network) into non-overlapping clusters or communities, sometimes called “network modules,” is an important way to explore functional roles of sets of genes. When the method to accomplish this decomposition is solely based on purely graph-theoretic measures of the interconnection structure of the network, this is often called *unsupervised* clustering or community detection. In this study, we compare unsupervised computational methods for decomposing a PPI network into non-overlapping modules. A method is preferred if it results in a large proportion of nodes being assigned to functionally meaningful modules, as measured by functional enrichment over terms from the Gene Ontology (GO).

**Results:**

We compare the performance of three popular community detection algorithms with the same algorithms run after the network is pre-processed by removing and reweighting based on the diffusion state distance (DSD) between pairs of nodes in the network. We call this “detangling” the network. In almost all cases, we find that detangling the network based on the DSD distance reweighting provides more meaningful clusters.

**Conclusions:**

Re-embedding using the DSD distance metric, before applying standard community detection algorithms, can assist in uncovering GO functionally enriched clusters in the yeast PPI network.

## Background

Clustering of protein-protein interaction networks is one of the most common approaches to predicting modules of genes and proteins that work together in functional roles [1]. However, the low network diameter and dense interconnection structure in these networks confounds a notion of local neighborhood in these networks; it is difficult to partition a network into clusters representing local neighborhoods when the network best resembles a tangled hairball, and most nodes are close to all other nodes in shortest path distance, a problem termed the “ties in proximity problem” by Arnau et al. [2]. There are nonetheless many notions of clustering that have been developed for the so-called “community detection” problem in biological or social networks; many of them seek to maximize the *modularity* of the clusters, a quantity defined by Girvan and Newman [3] that measures the relative denseness of interconnections within a cluster as compared to the connection of that cluster to the rest of the network, or alternatively the *conductance* of the clusters [4]. Other clustering methods have been proposed based on random walks, successive removal of cut edges, spectral embeddings and so on [5–7].

In 2013, Cao et al. introduced a new distance measure called Diffusion State Distance, or DSD, designed to be a more fine-grained distance measure for protein-protein interaction networks [8]. In contrast to the typical shortest path metric, which measures distance between pairs of nodes by the number of hops on the shortest path that joins them in the network, DSD was shown to spread out the pairwise distances, making for a more fine-grained notion of graph local neighborhood. We hypothesized that re-embedding the PPI network by first reweighting its edges according to their DSD distance in the original network might lead to better clusters. Before we can test this hypothesis, however, we need to think about how to measure the overall quality of a set of clusters: only then can we talk about once method producing *better* clusters than some other method.

### Measuring quality of a clustering

In the current study, we consider the problem of separating the yeast protein-protein association network (as downloaded from the STRING database [9]) into non-overlapping clusters. Some proposed ways to measure the quality of a clustering are purely graph-theoretic, based on minimizing quantities such as *modularity* or *conductance*. In this study, instead, we wish to judge the quality of the clustering we obtain by how “meaningful” the clusters are biologically– where the standard way to measure this would be based on measuring functional enrichment of the resulting clusters. In this study, we measure functional enrichment of the clusters over the GO using the FuncAssociate tool [10], with appropriate multiple testing correction for the number of clusters in our set. We declare a cluster to be functionally enriched if it is enriched for at least one and no more than 50 different GO terms, at an appropriate level of specificity in the GO hierarchy.

However, while it is easy to declare one particular cluster to be known to be meaningful if it is enriched for at least one and no more than 50 biological functions, it is not immediately clear how to use this to compare the overall quality of different clusterings, particularly when the number and distribution of cluster sizes is different across the different clustering algorithms. Observe that in particular, the *percentage of enriched clusters* is not a good statistic: any algorithm that picks off small good clusters around the periphery of the network, and then puts all the remaining nodes into a giant single cluster in the center, will score all but one of its clusters enriched (the large center cluster), for a very large percentage of enriched clusters. Restricting the maximum size of a cluster (as we do for some of the experiments) can ameliorate this behavior to a large extent, but we still are faced with the need to find a meaningful overall statistic even when the distribution of cluster sizes is highly non-comparable.

Because we are restricting ourselves to *non-overlapping* clusterings, we choose as the main statistic by which we judge the quality of a clustering to be *the number (or percent) of network nodes that are placed within enriched clusters.* We abreviate this as *#NEC* and *%NEC*. We note that this NEC statistic can be measured across clusterings with different numbers of clusters, size of clusters, and different cluster size distributions. However, even these NEC statistics are most meaningful when comparing clusterings when the number of clusters and their ranges of sizes are approximately matched; in particular, adding some number of unrelated nodes arbitrarily to an enriched clusters will improve the NEC statistics, even if it dilutes the cluster enrichment, as long as it doesn’t cause the enrichment to dip below the enrichment threshold. See Fig. 1 for a simple example demonstrating this case.

**Fig. 1:** Comparison of two example network partitions under the NEC statistic. Edges are omitted for visual clarity and only a single function *f* is considered in this simple case. The clusters outlined in bold blue are “enriched” and those outlined in dotted red are not. Although the lower partition is more specific for *f* (i.e. its enriched clusters contain fewer false positives), by the NEC statistic it does not score as well as the upper partition. Note that in this case, the distribution of cluster sizes is indeed much different between partitions; that is, the upper partition has a single giant cluster, and the lower partition contains clusters having a more uniform size distribution

Thus we add a second statistic that we call NEC S (for *number of enriched clusters, same label*), for the number (or percent) of nodes whose label *matches* a label of its enriched cluster. This is a more stringent condition met by a fewer number of nodes in enriched clusters and more precisely measures how well our clustering recapitulates exisiting knowledge. In the case where there is no bound on cluster sizes, this is the more meaningful statistic, because the ordinary NEC statistics will tend to inflate the quality of the clustering. Figure 2 shows the NEC S statistic computed on an example cluster.

**Fig. 2:** Example of scoring a single cluster using the NEC S statistic. GO annotations are listed for each node and for the cluster as a whole, and only those nodes with an annotation matching the cluster (the shaded nodes) are counted. In this case, 4 of the 6 total nodes (67%) are correctly clustered

Some of the algorithms we test allow greater or lesser control in setting maximum or minimum cluster sizes or the number of clusters that are output in the clustering; we discuss also how we would recommend setting these parameters in such a way as to make the resulting clusterings more meaningful for the biological networks we study, and also more comparable.

### The experiments

We implemented three popular methods for clustering biological or social networks in two modes: in the first mode, we ran them directly on the STRING network, and in the second mode, we first ran DSD to detangle the network, and then ran them on the network reweighted by edges inversely proportional to DSD distances. We considered each method in the setting where there was no restriction on maximum cluster size, and also in the setting where the maximum size of any cluster was bounded by 100 nodes. Some of the algorithms we test (such as Louvain) do not allow you to control for the *number* of clusters that our output; some of the algorithms give very fine control over this parameter. In order to make our results comparable across methods, we mainly focus on clusterings that produce between 200-300 clusters. In this range, when cluster sizes are bounded, we find that running DSD first to detangle the network results in a better percentage of nodes placed within enriched clusters. We note that when Walktrap modified to bound cluster sizes at 100 is run to output a large number of clusters, the results are more mixed: at 700 clusters, modified Walktrap performs better in the NEC statistic but slightly worse in the NEC S statistic when detangled with an appropriate DSD threshold, as compared to modified Walktrap run directly on the PPI network.

For the versions of the algorithm when maximum cluster size is unbounded, all algorithms perform better with detangling excepting spectral clustering with no bound on cluster sizes, where the performance is again mixed. For spectral clustering, a greater percentage of nodes in enriched clusters is produced when run directly on the PPI network, but the NEC S statistic (which is more meaningful when there is no bound on cluster sizes) is slightly better when DSD is run first. (When a bound of 100 nodes is again placed on maximum cluster size, performance by first detangling with DSD is again better by all measures).

We further discuss parameter settings that influenced the resulting number of clusters and their sizes in the network, and make recommendations for each method. In particular, we especially consider parameter settings where methods return between 200 and 300 clusters, each with between 3 and 100 nodes. In nearly all settings, we can advocate that re-weighting the network using DSD as a pre-processing step for decomposing protein-protein networks into functionally coherent communities produces more meaningful clusters.

## Review of DSD

Consider the undirected graph *G*(*V*,*E*) on the vertex set *V*={*v*_1_,*v*_2_,*v*_3_,...,*v*_*n*_} and |*V*|=*n*. Now *He*^{*k*}^(*A*,*B*) is defined as the expected number of times that a simple symmetric random walk starting at node *A* and proceeding for some fixed *k* steps (including the 0th step), will visit node *B*.

We now take a global view of the *He*^*k*^(*A*,*B*) measure from each vertex to all the other vertices of the network.

More specifically, we define a *n*-dimensional vector *He*^*k*^(*v*_*i*_),∀*v*_*i*_∈*V*, where

$$He^{k}(v_{i})=\left(He^{k}(v_{i}, v_{1}),He^{k}(v_{i}, v_{2}),...,He^{k}(v_{i}, v_{n})\right). $$

Then, the Diffusion State Distance (DSD) between two vertices *u* and *v*, ∀*u*,*v*∈*V* is defined as:

$$DSD^{k}(u,v)=\left\|He^{k}(u)-He^{k}(v)\right\|_{1}. $$

where ∥*He*^*k*^(*u*)−*He*^*k*^(*v*)∥_1_ denotes the *L*_1_ norm of the *He*^*k*^ vectors of *u* and *v*.

We showed in [8] for any fixed *k*, that DSD is a true distance metric, namely that it is symmetric, positive definite, and non-zero whenever *u*≠*v*, and it obeys the triangle inequality. Thus, one can use DSD to reason about distances in a network in a sound manner. Further, we show that when the network is ergodic, DSD converges as the *k* in *He*^{*k*}^(*A*,*B*) goes to infinity, allowing us to define DSD independent from the value *k*, and to compute the converged DSD matrix tractably, with an eigenvalue computation, where we can compute

$$DSD(u,v) = \left\|(1_{u} - 1_{v})\left(I- D^{-1}A + W\right)^{-1}\right\|_{1} $$

where *D* is the diagonal degree matrix, *A* is the adjacency matrix, and *W* is the constant matrix where each row is a copy of *π*, the degrees of each of the vertices, normalized by the sum of all the vertex degrees.

The above treatment does not consider edge weights; DSD was generalized to handle edge-weighted graphs in [11]. To incorporate edge weights, the random walk is modified where instead of choosing all edges at a vertex with equal probability, the walk instead chooses edges in proportion to their confidence weights, namely we define a new 1-step transition matrix with (*i*,*j*)th entry given by:

$$p'_{ij} = \frac{w_{ij}}{\sum_{l=1}^{n} w_{il}} $$

Then we redefine *He*^*k*^(*A*,*B*) as the expected number of times that the weighted random walk starting at node *A* and proceeding for *k* steps will visit *B*, which can be calculated as the (*i*,*j*)th entry of the *k*th power of the transition matrix. The *n*-dimensional vector *He*^*k*^(*v*_*i*_) can be constructed as before, and then the DSD is calculated the same as before, just based on the modified *He* vectors.

## Methods

### The network

The protein-protein association network for *S. cerevisiae* was downloaded from STRING version 10 on 2/7/2017 [9]. We removed all edges that had no direct experimental verification. Edge weights were taken directly from from the “escore” confidence values given by STRING. After we remove the 2 isolated nodes, the resulting network has 6096 nodes.

### Enrichment calculation

Functional enrichment was measured in Gene Ontology terms using the FuncAssociate 3.0 web API [10]. All GO terms that were level 5 or below in specificity from all three hierarchies (molecular function, biological process, and cellular component) were considered. FuncAssociate uses Fisher’s exact test to calculate an enrichment *p*-value, and we used a *p*-value cutoff of 0.05 to determine if a cluster was significantly enriched for a term. To correct for multiple testing, FuncAssociate uses an approach based on Monte Carlo sampling from the background gene space, as described in [10] (note that because of the stochastic sampling, different runs of FuncAssociate can give slightly different results, but we mostly observe differences of only fractions of a percentage point).

### The clustering algorithms

We considered the following popular clustering algorithms, each of which will return a non-overlapping set of clusters. In our study, we restricted cluster sizes to be at least 3; any cluster of size less than 3 created by an algorithm was discarded. We considered all three algorithms with no restriction on maximum cluster size; we then modified each of the three algorithms to set a maximum cluster size of 100. Bounds on minimum and maximum cluster size were set in order to make the clusterings returned by different methods more comparable; the specific values of 3 and 100 were set to be consistent with the recent DREAM community “disease module identification” challenge [12]. For each clustering method, we run it natively on the network from STRING. We then run it on a transformed network, preprocessed with DSD as follows: 1) We form the DSD matrix of distances in the original network. 2) We create a new graph by placing edges between pairs of nodes whose DSD distance is less than *r*, with edge weight 1/*r*. We then run the clustering algorithm on the new DSD-based detangled graph. We considered a range of different values of the threshold *r* (between 4 and 6).

#### The Louvain algorithm

For a partition of a network into two pieces, consider the quantity

$$Q =\frac{1}{2m}\sum_{i,j} \left[ A_{ij} - \frac{k_{i}k_{j}}{2m} \right] \delta(c_{i},c_{j}) $$

where *A*_*ij*_ is the matrix of edge weights, *m* is the sum of all the edge weights, $k_{i} = \sum _{j} A_{ij}$ is the sum of all the edge weights emanating from vertex *i* and *δ* is an indicator function that is 1 iff *i* and *j* have been placed in the same cluster. Then *Q* measures the *modularity* in a weighted graph, based on the weight of links within a cluster as compared to the links between clusters (see [3]).

The Louvain Algorithm, first defined in [13], is a heuristic that repeatedly tries to move individual nodes across cluster boundaries in order to improve the value of *Q*. Starting from a partition of the network into clusters (initially, every node is placed into its own cluster), the first phase of the Louvain algorithm considers nodes *i* that are adjacent to some node *j* which has been placed in a different community. *i* is moved into *j*’s community if and only if doing so would increase the modularity *Q* described above. Nodes are considered multiple times until the quantity *Q* can no longer be improved by moving any individual nodes. The second phase of the algorithm consists in building a new network whose nodes are now the communities found during the first phase. The weights between these new supernodes are now set to be the sum of the weight of the links between nodes in the corresponding two communities (where links between nodes of the same community are retained as self-loops). Then the first phase of the Louvain algorithm is run again on the new nodes.

In our implementation, clusters with less than 3 nodes were discarded. We also modified the Louvain algorithm to force clusters to have at most 100 nodes by re-running Louvain separately on each cluster with more than 100 nodes, in order to split the cluster into multiple clusters of size under 100 nodes.

#### The Walktrap algorithm

Consider the random walk on *G* where at each time step, the walker moves from a node to a new node chosen randomly and uniformly among its neighbors (in proportion to edge weights). When *D* is the matrix that has the *i*th diagonal entry be the degree of vertex *i*, and 0’s off the diagonal, then one can define the transition matrix of the random walk as *P*=*D*^−1^*A* where *A* is the adjacency matrix. Fix *t*, the length of a random walk and let $P^{t}_{i\circ }$ denote the *i*th row of the matrix *P*^*t*^ The Walktrap algorithm [14] defines an an (*i*,*j*) distance *r*_*i*,*j*_ depending on the *L*_2_ distance between the two probability distributions $P^{t}_{i\circ }$ and $P^{t}_{j\circ }$. This internode distance is then generalized to a distance between communities in a straightforward way, by choosing a starting node randomly and uniformly among the nodes of the community. This defines the probability $P^{t}_{C_{j}}$ to go from community *C* to vertex *j* in *t* steps and an associated probability vector $P^{t}_{C_{j}\circ }$. Then the distance $r_{C_{1}C_{2}}$ is defined as the *L*_2_ distance between the two probability distributions $P^{t}_{C_{1}\circ }$ and $P^{t}_{C_{2}\circ }$.

This algorithm is initialized by putting each vertex into its own cluster. Then two adjacent communities (joined by at least one edge) are merged according to which gives the lowest value of the quantity *Δα*, where the change in *Δα* that would result when clusters *C*_1_ and *C*_2_ are instead merged into a new cluster *C*_3_ is given by:

$$\Delta \alpha(C_{1}, C_{2}) = \frac{1}{n}\frac{|C_{1}||C_{2}|}{|C_{1}| + |C_{2}|} r^{2}_{C_{1}C_{2}} $$

In our implementation, we set *t*, the length of the random walk to 4, which is the recommended default. We discard all clusters of size < 3, and rerun replacing *t* with *t*−1 if any cluster remains of size > 100. The algorithm terminates when *t*=1, but Walktrap can still produce clusters of size > 100. We therefore also consider a modified version of Walktrap (again setting *t*=4) that prevents the merging clusters if the merge would create a cluster of of size >100. Modified Walktrap is run until no more merges are possible, which can be represented as a forest dendrogram (not a tree, because there are multiple clusters at the top level that cannot merge because their union would contain more than 100 nodes). We then cut the dendrogram at a lower level to produce some lower number of output clusters: the final number of clusters output is all the clusters at that level of size ≥ 3 (discarding clusters of size 1 or 2).

#### Spectral clustering

Spectral clustering was introduced by Ng, Jordan and Weiss [15] in 2001. It takes as input a similarity matrix, and does a low-dimensional embedding of the nodes according to that similarity matrix. Then *K*-means clustering is run on the nodes in the embedded space, where *K*, the number of clusters, is an input to the algorithm. In our case we construct the similarity matrix by computing 1/(the DSD distance). The final number of clusters we produce is not *K*, since we discard any cluster of size < 3. We consider also a modified version of spectral clustering where we recursively split any cluster of size > 100, recursively calling spectral clustering with *K*=2 clusters, until all cluster sizes are less than 100 nodes.

#### Clustering implementations

In the case of Louvain and unmodified Walktrap, we used the implementations in the popular igraph package [16]. In the case of spectral clustering, our implementation came from scikit-learn [17]. In the case of the modified Walktrap algorithm (which restricted cluster sizes to be < 100 nodes), we worked directly from the Walktrap source code from [14].

## Results

For each algorithm we consider, we compare what would be obtained by running that algorithm directly on the PPI network with weights taken directly from the STRING confidence values, with no filtering or pre-processing, to what is obtained by first running DSD on the network, filtering out edges where the DSD distance between their endpoints exceeded a threshold, and otherwise running the algorithm with edges weighted by 1/(DSD distance).

We first considered the Louvain and Walktrap algorithms without any restriction on maximum cluster size. The Louvain algorithm is highly sensitive to the order in which nodes are considered [13], so we report median results over 10 independent runs of the algorithm (mean results over the 10 runs are highly similar and not shown). The results appear in Tables 1 and 2. The best results occur when the network is pre-processed with DSD at an appropriate threshold, however, run directly on the PPI network as well as some of the DSD thresholds, these algorithms unmodified produce some large, uninformative clusters. For example, in every one of the 10 times we ran Louvain directly on the PPI network, the largest cluster had size greater than 1000 nodes. When we ran Walktrap directly on the PPI network, the largest cluster had size greater than 3000 nodes, i.e. nearly half the network was placed into a single, uninformative cluster. Thus we also considered modified versions of Louvain and Walktrap, as described above, that force cluster sizes between 3 and 100 nodes (where again, the specific values of 3 and 100 were set to be consistent with the recent DREAM community “disease module identification” challenge [12]). These results appear in Tables 3 and 4. DSD plus Louvain again performs better than Louvain alone, with bounded cluster sizes. However, Walktrap with bounded cluster sizes implemented directly on the PPI network seems to perform competitively (or even very slightly better) than DSD plus Walktrap with bounded cluster sizes. This was the one case of all the algorithms we tried where pre-processing the network using DSD did not clearly result in a superior quality clustering.

**Table 1:** The performance of Louvain run directly on the PPI network versus Louvain plus DSD at different edge removal thresholds; the reported results of Louvain are median values from running the algorithm over 10 random permutations of the nodes. We discard clusters of size < 3

Method	Enriched Clusters	# NEC	% NEC	# NEC S	% NEC S
PPI	29.5/47.5 (62.11%)	799.0	13.10%	548.5	8.99%
4.0	130.0/192.0 (67.71%)	1144.0	18.77%	1011.0	16.58%
4.5	175.0/265.5 (65.91%)	1960.5	**32.16%**	1562.0	**25.62%**
5.0	106.5/173.0 (61.56%)	1736.0	28.48%	967.0	15.86%
5.5	15.0/45.5 (32.97%)	361.5	5.93%	288.0	4.72%
6.0	5.0/21.5 (23.26%)	221.0	3.63%	178.5	2.93%

NEC= “Nodes in Enriched Clusters”. We calculate *%NEC* in two settings: *%NEC* is enrichment in the GO hierarchy with terms above the fifth level filtered out, and *%NEC* *S* uses the same filtered GO hierarchy, but then only gives a node credit if there is a match between one of the node’s labels and one of the terms for which there is GO enrichment for the cluster. Note that without modifying Louvain to restrict the maximum cluster size, the *S* statistic is the most meaningful. Running directly on the PPI network and run with high DSD thresholds, Louvain produces a relatively small number of clusters, and many are of very large size. It is worth noting that with a DSD threshold of 5, nearly 175 clusters are produced, and the enrichment statistics remain reasonable

Bolded values represent the best values achieved for the *%NEC* and *%NEC* S statistics comparing the PPI network and different DSD detangling thresholds

**Table 2:** The performance of Walktrap versus Walktrap plus DSD at different edge removal thresholds; We discard clusters of size < 3

Method	Enriched Clusters	# NEC	% NEC	# NEC S	% NEC S
PPI	8/19 (42.11%)	280.0	4.59%	226.0	3.71%
3.5	63/105 (60.00%)	504.0	8.27%	464.0	7.61%
4.0	128/189 (67.72%)	1108.0	18.18%	919.0	15.08%
4.5	207/311 (66.56%)	1951.0	32.00%	1430.0	23.46%
5.0	153/303 (50.50%)	2476.0	**40.62%**	1531.0	**25.11%**
5.5	70/164 (42.68%)	2418.0	39.67%	1269.0	20.82%
6.0	43/88 (48.86%)	1398.0	22.93%	837.0	13.73%

NEC= “Nodes in Enriched Clusters”. We calculate *%NEC* in two settings: *%NEC* is enrichment in the GO hierarchy with terms above the fifth level filtered out, and *%NEC* *S* uses the same filtered GO hierarchy, but then only gives a node credit if there is a match between one of the node’s labels and one of the terms for which there is GO enrichment for the cluster. Walktrap run alone produces a very small number of clusters; because of this only the *S* statistic is meaningful to compare the DSD versions against unmodified Walktrap. Walktrap with DSD at thresholds between 4.5 and 6 trade a larger number of smaller clusters for a lower percentage of nodes in enriched clusters

Bolded values represent the best values achieved for the *%NEC* and *%NEC* S statistics comparing the PPI network and different DSD detangling thresholds

**Table 3:** The performance of Louvain versus Louvain plus DSD at different edge removal thresholds; the results of Louvain are median values from running the algorithm over 10 random permutations of the nodes. We discard clusters of size < 3 and prevent combining clusters when the resulting cluster would have size > 100

Method	Enriched Clusters	# NEC	**% NEC**	# NEC S	**% NEC S**
PPI	78.0/382.0 (20.42%)	1543.5	25.31%	634.5	10.41%
4.0	130.0/192.5 (67.53%)	1138.0	18.67%	1007.0	16.52%
4.5	186.0/305.0 (60.98%)	1915.5	31.42%	1297.5	**21.28%**
5.0	137.0/352.0 (38.92%)	2283.5	**37.46%**	1017.5	16.69%
5.5	53.5/227.5 (23.52%)	1987.0	32.60%	462.5	7.59%
6.0	40.5/180.5 (22.44%)	1702.5	27.93%	317.5	5.21%

NEC= “Nodes in Enriched Clusters”. We calculate *%NEC* in two settings: *%NEC* is enrichment in the GO hierarchy with terms above the fifth level filtered out, and *%NEC* *S* uses the same filtered GO hierarchy, but then only gives a node credit if there is a match between one of the node’s labels and one of the terms for which there is GO enrichment for the cluster. At every DSD threshold we tested except 4, the percentage of nodes in enriched clusters is better than Louvain run alone. The *S* statistic is better at DSD thresholds between 4 and 5, and best at a DSD threshold of 4.5

Bolded values represent the best values achieved for the *%NEC* and *%NEC* S statistics comparing the PPI network and different DSD detangling thresholds

**Table 4:** The performance of Modified Walktrap versus Modified Walktrap plus DSD at different edge removal thresholds; We discard clusters of size < 3, and restrict maximum cluster size to be < 100

Method	Enriched Clusters	# NEC	% NEC	# NEC S	% NEC S
PPI	35/64 (54.69%)	3274.0	53.69%	1703.0	27.93%
3.5	56/91 (61.54%)	570.0	9.35%	468.0	7.68%
4.0	97/142 (68.31%)	1155.0	18.95%	915.0	15.01%
4.5	144/215 (66.98%)	1869.0	30.66%	1415.0	23.21%
5.0	96/174 (55.17%)	2785.0	45.69%	1724.0	28.28%
5.5	56/93 (60.22%)	4067.0	66.72%	1783.0	**29.25%**
6.0	51/81 (62.96%)	4155.0	**68.16%**	1667.0	27.35%
PPI	39/69 (56.52%)	3367.0	55.21%	1782.0	29.22%
3.5	55/91 (60.44%)	495.0	8.12%	463.0	7.60%
4.0	97/142 (68.31%)	1155.0	18.95%	915.0	15.01%
4.5	144/215 (66.98%)	1869.0	30.66%	1415.0	23.21%
5.0	95/174 (54.60%)	2686.0	44.06%	1676.0	27.49%
5.5	60/106 (56.60%)	3978.0	65.26%	1862.0	**30.54%**
6.0	66/96 (68.75%)	4077.0	**66.88%**	1680.0	27.56%

The numbers above the double line are for cutting the Walktrap dendrogram at 200 clusters; the numbers below the double line are for cutting the Walktrap dendrogram at 300 clusters. NEC= “Nodes in Enriched Clusters”. We calculate *%NEC* in two settings: *%NEC* is enrichment in the GO hierarchy with terms above the fifth level filtered out, and *%NEC* *S* uses the same filtered GO hierarchy, but then only gives a node credit if there is a match between one of the node’s labels and one of the terms for which there is GO enrichment for the cluster. In both cases, for the *S* statistic the best DSD threshold is 5.5, at which performance is slightly better than running Walktrap directly on the PPI network. For cutoffs of both 200 and 300 nodes, DSD+Walktrap is slightly better than Walktrap in the *NEC* measure, and in both cases the DSD version produces slightly more and smaller clusters

Bolded values represent the best values achieved for the *%NEC* and *%NEC* S statistics comparing the PPI network and different DSD detangling thresholds

In order to explore our chosen measure of cluster quality, namely, the percent of the 6096 network nodes placed into an enriched cluster of size between 3 and 100 further, for Walktrap modified to have bounded cluster size run directly on the PPI network versus run after pre-processing with various DSD thresholds, we explored cutting the Modified Walktrap dendrogram at different numbers of clusters (before filtering small clusters, so the resulting numbers of clusters may not necessarily be exactly the same as the dendrogram cut level). The results appear in Tables 5 and 6, for both the *%NEC* and *%NEC* *S* statistics. For the *%NEC* statistic, the modified Walktrap algorithm with DSD preprocessing performs better for every dendrogram cut level. For the *%NEC* *S* statistic, the algorithm with DSD preprocessing performs better for lower dendrogram cut levels (i.e. fewer clusters), but for a dendrogram cut level of 700, the algorithm run directly on the PPI network performs better, although DSD with a cutoff of 5.5 performs comparably for this statistic.

**Table 5:** Exploring the dendrogram cut level for modified Walktrap with a maximum cluster size of 100

Dendrogram cut level	200	300	500	700
PPI	55.3%	53.6%	54.9%	55.3%
DSD 4.5	30.7%	30.7%	30.7%	30.3%
DSD 5	44.1%	44.0%	44.1%	44.2%
DSD 5.5	66.7%	66.9%	65.1%	**65.3%**
DSD 6	**72.6%**	68.3%	**66.2%**	63.0%
DSD 6.5	65.5%	**68.4%**	61.8%	53.7%

The reported number is the percentage of nodes placed into an enriched cluster (i.e. the statistic we are calling % NEC). At different dendrogram cut levels, the best percentage is bolded; in every case it is modified Walktrap plus DSD, at varying thresholds (5.5, 6, and 6.5)

**Table 6:** Exploring the dendrogram cut level for modified Walktrap with a maximum cluster size of 100

Dendrogram cut level	200	300	500	700
PPI	29.0%	28.0%	30.2%	**32.3%**
DSD 4.5	23.3%	23.2%	23.2%	24.5%
DSD 5	27.3%	27.5%	27.4%	28.9%
DSD 5.5	**29.6%**	**31.5%**	**30.6%**	31.8%
DSD 6	28.4%	27.8%	27.5%	24.8%
DSD 6.5	25.0%	26.9%	23.6%	19.9%

The reported number is the percentage of nodes placed into a cluster with a matching annotation (i.e. the statistic we are calling % NEC S). At different dendrogram cut levels, the best percentage is bolded; sometimes it is modified Walktrap run directly on the PPI network, and sometimes it is Walktrap plus DSD at a threshold of 5.5

Figure 3 gives some intuition for how the DSD thresholds were chosen: it shows a histogram of all pairwise DSD distances between nodes in the PPI network; setting the DSD threshold removes a fraction of these edges and sparsifies the network. For example, setting the edge removal threshold to 4.5 will result in direct edges from a vertex only to a small fraction of its close neighbors in DSD distance. Setting the edge removal threshold to 6, on the other hand, preserves roughly half the pairwise network distances.

**Fig. 3:** Histogram of all DSD distances in the STRING PPI network for yeast; edge removal thresholds of 4.5 and 6.0 are marked

Figure 4 directly compares the clusters at different size ranges by enrichment for Louvain directly, and DSD followed by Louvain, with an edge removal threshold of 5, and cluster sizes bounded to lie between 3 and 100. Detangling with DSD increases the percentage of nodes placed within enriched clusters. Figure 5 directly compares the clusters at different size ranges by enrichment for Walktrap directly, and DSD followed by Walktrap, with an edge removal threshold of 5.5, and cluster sizes bounded to lie between 3 and 100. In this case, the two clusterings are actually quite comparable in terms of the percentage of nodes placed within enriched clusters, but without the DSD detangling, the algorithm creates a greater number of larger clusters.

**Fig. 4:** This figure compares median cluster sizes running Louvain (with cluster sizes restricted to 3-100) directly on the PPI network with Louvain running on the DSD-detangled network (again with cluster sizes restricted to 3-100), with an edge removal threshold of 5.0. The overall percentage of nodes in enriched clusters is 25.31% for Louvain directly and 37.46% for DSD+Louvain

**Fig. 5:** This figure compares cluster sizes running Walktrap (with cluster sizes restricted to 3-100) directly on the PPI network with Walktrap running on the DSD-detangled network (again with cluster sizes restricted to 3-100), with an edge removal threshold of 5.5, using a dendrogram cutoff of 300. The percentage of nodes in enriched clusters is 55.21% for Walktrap directly and 65.26% for DSD+Walktrap

We next sought to make the comparison for spectral clustering, but spectral clustering has an additional parameter that must be set, namely *K*, the number of clusters. We look at both a version of spectral clustering that does not restrict maximum cluster size, as well as a variant of spectral clustering that recursively splits clusters of size greater than 100, in order to produce a clustering with clusters of size between 3 and 100 nodes, as before. Note that the final number of clusters output by our spectral clustering method will be different than *K*, the input number of cluster centers, because our implementation of spectral clustering recursively splits any cluster of size > 100. Figure 6 shows that the number of clusters that spectral clustering plus DSD (modified to force a maximum cluster size of 100) produces based on the number of input clusters is robust to the threshold cutoff. In all cases, the number of output clusters rises for awhile based on the number of input cluster centers, and then falls off. It rises compared to the number of input clusters when cluster sizes are too large and get split by our method for having > 100 nodes. It falls off when *K* is set large enough that many of the clusters that spectral clustering produces have < 3 nodes, which we then discard and do not include as output clusters according to the cluster size restrictions of our methods. Based on this figure, we report results for *K*=300 at different DSD thresholds in Tables 7 and 8.

**Fig. 6:** This figure plots the number of clusters output by spectral clustering and spectral clustering run on the DSD reweighted network, for different filter distance thresholds, based on the number *K* of clusters input to the method; in all cases, the number of output clusters starts out as less than *K* since clusters of size < 3 are not included in the count of output clusters. Then the number of clusters grows larger than the number of input clusters (because large clusters are recursively split) until *K* grows so large that the number of clusters of size < 3 counterbalances that increase

**Table 7:** The performance of Spectral versus Spectral plus DSD at different edge removal thresholds when the input parameter *K* in all cases is set to 300, but then we discard clusters of size < 3

Method	Enriched Clusters	# NEC	% NEC	# NEC S	% NEC S
PPI	201/225 (89.33%)	5650.0	**92.65%**	2409.0	39.50%
4.5	185/244 (75.82%)	2190.0	35.93%	1322.0	21.69%
5.0	176/252 (69.84%)	5003.0	82.07%	2100.0	34.45%
5.5	175/251 (69.72%)	4651.0	76.30%	2223.0	36.47%
6.0	168/224 (75.00%)	4997.0	81.97%	2473.0	**40.57%**

NEC= “Nodes in Enriched Clusters”. We calculate *%NEC* in two settings: *%NEC* is enrichment in the GO hierarchy with terms above the fifth level filtered out, and *%NEC* *S* uses the same filtered GO hierarchy, but then only gives a node credit if there is a match between one of the node’s labels and one of the terms for which there is GO enrichment for the cluster. In this case, the Spectral algorithm run directly on the PPI network results in a higher *%NEC* statistic than any of the DSD-preprocessed results. However, without cluster size restrictions *%NEC* *S* is the most meaningful statistic, and it is better than Spectral run alone at a DSD threshold of 6.0

Bolded values represent the best values achieved for the *%NEC* and *%NEC* S statistics comparing the PPI network and different DSD detangling thresholds

**Table 8:** The performance of Spectral versus Spectral plus DSD at different edge removal thresholds when the input parameter *K* in all cases is set to 300, but then we discard clusters of size < 3 and split clusters of size > 100

Method	Enriched Clusters	# NEC	% NEC	# NEC S	% NEC S
PPI	234/324 (72.22%)	3082.0	50.54%	2158.0	35.39%
4.5	194/266 (72.93%)	1647.0	27.02%	1330.0	21.82%
5.0	199/309 (64.40%)	3589.0	58.87%	2203.0	36.14%
5.5	189/291 (64.95%)	3765.0	61.76%	2228.0	36.55%
6.0	177/249 (71.08%)	4670.0	**76.61%**	2490.0	**40.85%**

NEC= “Nodes in Enriched Clusters”. We calculate *%NEC* in two settings: *%NEC* is enrichment in the GO hierarchy with terms above the fifth level filtered out, and *%NEC* *S* uses the same filtered GO hierarchy, but then only gives a node credit if there is a match between one of the node’s labels and one of the terms for which there is GO enrichment for the cluster. For every threshold we tested ≥ 5, the percentage of nodes in enriched clusters is better than Spectral run alone for both measures

Bolded values represent the best values achieved for the *%NEC* and *%NEC* S statistics comparing the PPI network and different DSD detangling thresholds

Figure 7 gives the number of clusters and the percentage of enriched clusters for spectral clustering (with a maximum cluster size bounded at 100) and DSD+spectral clustering for *K*=300. As can be seen, DSD+spectral clustering has a higher percentage of nodes in enriched clusters than spectral clustering alone.

**Fig. 7:** This figure compares cluster sizes running Spectral (with cluster sizes restricted to 3-100) directly on the PPI network with Spectral running on the DSD-detangled network (again with cluster sizes restricted to 3-100), with an edge removal threshold of 5.5. The percentage of nodes in enriched clusters is 50.54% for Spectral directly and 61.76% for DSD+Spectral

## Discussion

It is hard to definitively answer which of the six methods we tested is best, since it is hard to control the range of cluster sizes exactly. Clearly, the Louvain algorithm is performing worse in our setting than Walktrap or spectral clustering. In fact, spectral clustering plus DSD is able to produce an impressive percent of nodes in enriched clusters, in a setting where it is very easy to control the number and size range of the clusters that are returned. For this reason, the spectral clustering method was probably our favorite, though modified Walktrap also performed quite well, both with and without DSD.

Measuring the number of nodes placed into enriched clusters (not necessarily enriched for their own label) showed similar trends regardless of whether or not we filtered out the most general GO terms; these statistics were also often improved at the appropriate DSD threshold when sizes and and number of clusters were approximately matched.

It is natural to ask if our results were peculiar to the yeast network, or whether they would generalize to other organisms. We were particularly interested in the human network, which has more nodes but is more sparsely annotated. We thus also downloaded the protein-protein interaction network for *H. sapiens* from STRING version 10 on 2/7/2017. As before, we removed all edges that had no direct experimental verification. Edge weights were taken directly from the ’escore’ confidence values given by STRING. In the human network, we consider only the largest connected component which has 15,129 nodes.

Because there are fewer known edges and this is a sparser network than yeast, we set higher DSD thresholds, ranging from 6 to 8. See Fig. 8 for the corresponding histogram of all pairwise DSD distances in this network.

**Fig. 8:** Histogram of all DSD distances in the Human STRING PPI network; previous edge removal thresholds of 4.5 and 6.0 for yeast are marked

As can be seen in Table 9, the advantages of detangling the network with DSD before applying Spectral clustering seem even clearer on the human network. For both of the *%NEC* thresholds, and robust to the exact value of the DSD cutoff, results are better when the network is pre-processed with DSD.

**Table 9:** The performance of Spectral versus Spectral plus DSD at different edge removal thresholds when the input parameter *K* in all cases is set to 300, but then we discard clusters of size < 3 and split clusters of size > 100 on the Human network

Method	Enriched Clusters	# NEC	% NEC	# NEC S	% NEC S
PPI	252/510 (49.41%)	4540.0	29.96%	2301.0	15.18%
6.0	268/543 (49.36%)	6632.0	43.84%	2453.0	16.21%
6.5	286/543 (52.67%)	7085.0	46.83%	2918.0	19.29%
7.0	269/537 (50.09%)	7485.0	49.47%	3092.0	20.44%
7.5	272/552 (49.28%)	7243.0	47.87%	3073.0	20.31%
8.0	268/491 (54.58%)	7689.0	**50.82%**	3208.0	**21.20%**

We calculate *%NEC* in two settings: *%NEC* is enrichment in the GO hierarchy with terms above the fifth level filtered out, and *%NEC* *S* uses the same filtered GO hierarchy, but then only gives a node credit if there is a match between one of the node’s labels and one of the terms for which there is GO enrichment for the cluster. By both of the NEC statistics, at every DSD threshold, detangling with DSD performs better

Bolded values represent the best values achieved for the *%NEC* and *%NEC* S statistics comparing the PPI network and different DSD detangling thresholds

Many open questions still remain. In future work, we will measure whether a similar DSD pre-processing step improves algorithms for overlapping community detection in other biological networks. We will verify that we get similar results on networks arising from additional species, and also seek to investigate whether the results remain true on networks built using different types of gene-gene or protein-protein association data. We will continue to study the best way to measure cluster quality when faced with a different number of clusters of different sizes. Finally, one way in which our problem formulation was somewhat artificial is that we required our clusters to be *non-overlapping*; however, many proteins participate in multiple pathways, complexes or processes, which would be more accurately represented by overlapping clusters or communities. A recent survey of methods for overlapping community detection appears in [18].

## Conclusion

We have shown that some popular network community detection methods appear to perform better at identifying functionally enriched clusters when DSD is applied as a pre-processing step to help detangle the network. In particular, we tested the Louvain, Walktrap and Spectral Clustering methods, both native as well as modified to keep the maximum cluster size bounded by 100 nodes. Each method was run on the yeast PPI network directly, and then run on the PPI network after using DSD to sparsify and detangle the network.

For five of the six methods, applying the DSD pre-processing method at an appropriate threshold improved the percentage of network nodes that were placed into clusters enriched for their own functional label. For the sixth method, spectral clustering with no modification to large clusters, the DSD detangling sometimes improved performance slightly or sometimes hurt performance slightly, depending on other parameter settings.
